The article "Changes of Substance P in the Crevicular Fluid in relation to Orthodontic Movement Preliminary Investigation" was published in 2013. Journal: ScientificWorldJournal.

# Changes of Substance P in the Crevicular Fluid in relation to Orthodontic Movement Preliminary Investigation

**DOI:** 10.1155/2013/896874

**Published:** 2013-04-23

**Authors:** Luca Levrini, Paola Sacerdote, Sarah Moretti, Silvia Panzi, Alberto Caprioglio

**Affiliations:** ^1^Dipartimento di Scenze Chirugiche e Morfologiche, Università degli Studi dell'Insubria, 2110 Varese, Italy; ^2^Dipartimento di Scienze Farmacologiche e Biomolecolari, Università degli Studi di Milano, 20129 Milano, Italy

## Abstract

Substance P (SP) is a tachykinin released from both the central and the peripheral endings of primary afferent neurons and functions as a neurotransmitter. As a transmitter signaling pain, substance P is involved in nociception and is an extremely potent vasodilator. We found several studies about this neuropeptide especially in relation to parodontology and a few orthodontic reviews. This is because in the past the importance of this neuropeptide in dental element undergoing periodontal inflammation was observed. The aims of the present pilot study was to investigate whether the substance P was present in gingival crevicular fluid in dental elements undergoing orthodontic treatment with Invisalign technique compared to teeth belonging to the same series but not undergoing orthodontic movement. We analysed gengival crevicular fluid (GCF) collected from four young subjects, using a paper cone for a time of 60 seconds. The results showed that SP is present in the gengival sulcus in elements undergoing orthodontic forces during treatment with Invisalign technique and not in the control teeth. During the literature analysis, we have found a lot of papers describing involvement of SP in periodontitis and inflammatory diseases, but further studies are needed in order to demonstrate the role of this neuropeptide during teeth movement.

## 1. Introduction

The mechanical stress applied to a tooth due to orthodontic treatment induces an inflammatory reaction which leads to the remodelling of periodontal tissues, resulting in tooth movement. Since the periodontal ligament (PDL) and the dental pulp are well innervated and contain numerous receptors for noxious stimuli, it is conceivable that neurotransmitters, in particular substance P, could mediate the biological response to mechanical stress applied to the teeth during orthodontic treatment [1]. It is clear from the literature [2] that all orthodontic procedures such as the use of elastic separators [3], the placement of braces, and the application of orthopaedic forces cause pain in patients. It is also known that nonremovable devices produce more pain than removable or functional devices and there is a poor correlation between the intensity of the applied force and the pain experienced. The experiences reported by many patients after placement of the device are often described as sensations of pressure, tension, and teeth pain. There is no demonstrated relationship between age, sex, and psychological and cultural perception of pain following the placement of an orthodontic appliance. The correlation between the psychological well-being of patients and the perception of orthodontic pain was proved without doubt. We know from the published literature that women feel more pain than men, and adolescents report higher levels of pain than preteens and adults [1]. Substance P is a neuropeptide known to be deputed to nociceptive transmission signal [4–6]. The history of this molecule began in 1931 when scholars Von Euler and Gaddum isolated the substance from the brain and intestine of horses. Several studies [7] have stressed the importance of substance P as a mediator of pain and inflammation. In particular, we can observe an increase in the concentration of the neuropeptide in the pulp of patients suffering from caries, pulpitis, and granulomas and during movement of the dental elements consequent to orthodontic treatment [7]. Substance P is present in the sulcular fluid; from this drawing its concentration is assessable. The purpose of this pilot study was to verify the experimental feasibility and observe the change in the concentration of substance P in dental elements undergoing orthodontic forces during treatment with Invisalign technique. The choice of this type of device was due to the need of something that can predict the presence or absence of tooth movement. Different studies have already analyzed the different concentrations of SP, comparing different multiband systems, with the aim to reduce inflammation and pain [8, 9]. Main articles were identified by a specific search MEDLINE using appropriate keywords (e.g., substance P and dental movement or orthodontic movement), which was then refined manually browsing the reference lists of articles retrieved and with the addition of other relevant documents according to the authors' knowledge of the field. 

### 1.1. Teeth Movement

Each tooth is attached to the surrounding alveolar bone and at the same time separated from it by a robust support structure of collagen: the periodontal ligament (PDL). Its main component is represented by a set of parallel collagen fibers which are placed between cement and a relatively robust bone surface: the lamina dura. The space of the PDL (about 0.5 mm) is occupied by the tangle of fibers, but there are two other important components of the periodontal ligament: the cellular component consists of a variety of mesenchymal cells and tissue fluids. Although not intensely vascularized, the PDL has vessels and cells of the blood system. There are also unmyelinated nerve fibers, appointed to the perception of pain and complex receptor associated with the pressure and proprioceptive information [10–12]. During normal chewing, teeth and periodontal structures are subject to heavy forces [13] and intermittent, ranging from 1 to 2 kg when you chew soft foods that can reach up to 50 kg for harder foods. When the tooth is subjected to loads of this type, its rapid displacement in space of the PDL is prevented by the presence of the fluid, by its nature incompressible. The force is transmitted thereby to the walls of the alveolar process, causing a deflexion of the support structures, often not appreciable. Only a small part of the fluid, contained in the space of the PDL, is ejected during the first second of solicitation pressure. However, if the pressure will be maintained on the tooth, this fluid may be expelled and the tooth is moved in space of the PDL, in turn compressed against the walls adjacent bone. The pain will normally be perceived in 3–5 seconds after application of a heavy force, a sign that the liquid was squeezed out. Tooth movement induced by application of orthodontic forces (orthodontic tooth movement (MDO)) is based on the remodelling of the dental and periodontal tissues [14]. Two interrelated processes involved in MDO are flexion of the alveolar bone and remodelling of periodontal tissues, including dental pulp, periodontal ligament (PDL), the alveolar bone, and the gum [15]. When we apply a continuous and light force to the tooth, we can observe a reduction of blood flow through the PDL partially compressed; this occurs as soon as the fluids are pushed outside the periodontal space following the displacement of the tooth in the alveolar bone (in a few seconds). Within a few hours, the chemical changes occurred induce a different model of cellular activity. In animal experiments, increased levels of adenosine 3′, 5′ monophosphate (cAMP), the “second messenger” of many functions involved in cellular differentiation, were found; this occurs approximately 4 hours after the application of continued pressure [16]. The same amount of time was necessary in humans to get a first response to the application of removable devices. In fact, if these devices are worn for less than 4–6 hours a day, they will not induce any orthodontic effect [17]. 

## 2. Materials and Methods

The sample examined consisted of all the subjects treated with Invisalign technique at the Dental Clinic of the University of Insubria. Among these, through the analysis of the ClinCheck Invisalign (Figure 1), four patients were chosen where the tooth movement to be achieved was a simple flaring that was an inclination of a degree of the dental element to the fornix (Figure 2), considering the long axis as a guide to the movement (experimental sample); at the same time there had to be an element in the same dental arch and contralateral without movement (control sample). Three of these couples were in the incisors series, three belonged to premolar, and two molars. Among these four young female patients were selected aged respectively 13 years and 10 months–19 years and 11 months–17 years and 6 months and 15 years and 7 months, with a molar ratio of first class, canine ratio of first class. It was also verified that the subjects examined showed (1) a general good health, (2) the lack of antibiotic therapy in the past six months, (3) no use of anti-inflammatory drugs during the month preceding the study, (4) periodontal health with generalized and physiological probing depth of 2 mm, (5) no radiographic evidence of bone loss, (6) crowding in one or both jaws, (7) a bleeding index of zero, and (8) absence of caries and tartar. Informed consent was obtained from the patients and parents before the study. Before the beginning of therapy, all patients had an appointment of oral hygiene with ultrasonic instruments. Probing depth, presence of plaque, and bleeding were evaluated on both arches. The drawings (Figure 2) were performed both on the dental element that would have been the subject of orthodontic force compressed by the movement of flaring and on the motionless one. The sites selected for GCF sampling were isolated using cotton wool rolls and a saliva ejector. Supragingival plaque was carefully removed using a curette. We took four samples from one subject probing depth from the four lower incisors (element 3.2 and 4.1 were test and 3.1 and 4.2 control). From the second patient we analysed six elements from premolar series (elements 1.4 and 1.5 and 4.5 as control, elements 2.4, 2.5, and 3.4 as test) and two elements from the molar series (4.6 as control and 3.6 as test). From patient three, we studied two elements from the molar series (1.6 as test and 2.6 as control). From patient four, we analysed two elements from incisors series (3.2 as test and 3.1 as control). Before introducing the paper cone (Periopaper, Harco, Tustin, CA, USA), in the gingival sulcus, it has been dried with warm air for 10 seconds. The instrument was introduced, taking care to avoid mechanical damage, for a time of 60 seconds always in the mesial portion of element. The drawing of sulcular fluid was carried out using paper cones with a diameter of 35 × 10^−5^ m (Figure 3). The cones were introduced in the gingival sulcus of the element for a time of thirty seconds and then stored in a fridge at −30°C. Elution of SP from each paper strip was performed by centrifugation of the samples in 0.4 mL of 0.02 M Tris-HCL buffer (pH 7.5) for 30 minutes, and the supernatant was collected for SP measurement [18]. The amount of SP in each sample was determined by enzyme linked immunosorbent assay (ELISA) with a commercially available kit (R & D Systems, Minneapolis, MN, USA). The results are expressed as the total amount per 60 s GCF samples. 

## 3. Results

The average value of SP concentration in the GCF drawings obtained from the experimental samples was 13.4 pg ± 6.8 (mean ± SD), while that of the control group was 4.2 pg ± 0.6 (Table 1). The levels of SP detected in control elements were always very low at the limit of detection. The teeth movement increased the levels of the neuropeptide in all patients. Statistical evaluation of results with Student's *t*-test showed the presence of a significant difference between experimental samples and controls (*P* < 0.01).

## 4. Discussion

Recently the role of SP in the modulation of pain and inflammation in dental procedures has attracted much attention. However the studies examining the modulation of this neuropeptide in orthodontic movements are still scarce. Although we are aware of the limited number of patients in our pilot study, the data obtained seem to confirm an involvement of SP during this type of procedures. In particular our pilot study is the first study to examine the SP concentration in the GCF after the Invisalign procedure. Interestingly a recent study carried out by Miller et al. [19] has shown that adults treated with Invisalign aligners felt less pain and fewer negative impacts on their lives during the first week of orthodontic treatment compared to those treated with fixed appliances. In this prospective longitudinal study carried out on 60 adult orthodontic patients (33 with Invisalign aligners, 27 with fixed appliances), pain was assessed using a daily diary to measure the impact of treatment in terms of functional, psychosocial, and pain related results. A diary was completed for seven consecutive days in order to measure the impact of orthodontic treatment. The baseline mean values did not differ between groups for pain reports or overall quality of life impact. During the first week of treatment, the subjects in the Invisalign group reported fewer negative impacts on overall quality of life. The Invisalign group also recorded less impact in each quality of life subscale evaluated (functional, psychosocial, and pain-related). The visual analog scale pain reports showed that subjects in the Invisalign group experienced less pain during the first week of treatment. The subjects in the fixed appliance group took more pain medications than those in the Invisalign group at days 2 and 3. Yamaguchi et al. demonstrated that the levels of SP and IL-1 in GCF are increased by orthodontic movement [9]. The study was carried out by Yamaguchi et al. [9], by using Damon's technique. They showed that there was no significant difference in respect to the control site in the mean volume of SP during the therapy between the groups where conventional braces were utilized comparing to self-ligating attachment and the control site [20]. The same authors [18] analysed nine adult orthodontic patients treated with fix appliance. The experimental protocol provided the extraction of a first premolar in order to allow the canine distalization (with an elastic chain) and use the contralateral element as a control group. The samples SP performed after 8, 24, and 72 hours showed a higher concentration of substance P in the test site than the control, while the samples carried out at 168 hours showed that the SP value was lower in the test site than control. Nicolay and colleagues [1] hypothesized that the SP could mediate the biological response of the mechanical stress applied to the teeth during orthodontic treatment and performed a study in the cat using an immunohistochemical technique. They applied a force, for a time ranging from 1 hour to 14 days, using a group of cats tipping distally the maxillary canine. Horizontal histological sections, 5 *μ*m thick, collected from frozen specimens were stained using rabbit anti-SP polyclonal antibodies. This preliminary study showed that the stimulation of periodontal nerve fibers by means of orthodontic forces may induce peripheral release of SP in the pulp and PDL. The SP may be the initial trigger for a biochemical cascade that leads to the activation of target cells in the periodontium. SP can either act directly on the target cells as a “first messenger” or enhance the release of other messengers as prostaglandins and cytokines, leading to an increase of “intracellular second messengers.” In both cases, the SP appears to play a key role in the regulation of cellular responses to mechanical forces in vivo. A higher number of studies have evaluated the levels of SP and SP-related peptides in several oral diseases such as periodontitis and pulp inflammation. Awawdeh and colleagues [21] evaluated 20 patients, half of which were affected by periodontal disease, the concentrations of SP and neurokinin A (NKA). Gingival crevicular fluid (GCF) was collected from 20 subjects in three different sites: the first was a healthy site, the second presented gingivitis, and the third periodontitis. The aim of the study was to investigate whether the substance P and neurokinin A were present in gingival crevicular fluid in both periodontal health and disease and to study the relationship with periodontal inflammation. In subjects with periodontitis, there were significant increases in the levels of SP and NKA in both sites with periodontal disease in comparison to healthy sites. Interestingly subjects with periodontitis showed increased levels of SP also in healthy sites, when compared with patients without periodontal disease. Similar results were found by Alstergren et al. [22], in fluid aspirated from temporomandibular joints. The higher levels of substance P in GCF particularly in diseased sites may indicate that SP has a more important role in periodontal inflammation than NKA. In fact Pernow [23] reported that the proinflammatory potency of SP is greater than NKA. The proinflammatory effects of tachykinins may, however, be counterbalanced by their reparative and regulatory roles that have only recently been elucidated. SP and NKA stimulate DNA synthesis when added to cultured skin fibroblasts [24]. Bartold et al. [25] have shown that SP can influence human gingival fibroblast proliferative and synthetic activity and suggested that the action of this peptide could switch from a catabolic proinflammatory mode to an anabolic tissue regenerative mode depending on the presence of other factors. Tachykinins released by peripheral neurones could not only contribute to the inflammatory response, but also act to stimulate proliferation of surrounding connective tissue cells starting a healing response in tissue. SP and NKA may have a relationship with periodontal disease. A systematic study of the relationship of these tachykinins and other neuropeptides in periodontal disease may be useful for further clarifying the mechanisms that regulate the health and periodontal disease. Hanioka and colleagues [18] observed 48 subjects with periodontal disease at an advanced stage, with gingival inflammation and shallow or moderately deep pocket. Gingival crevicular fluid was collected at one site per subject from the mesial surface of the palatal aspect of maxillary canines or premolars. The experimental site was selected according to the worst score of gingival inflammation. The level of inflammation and destruction of the supporting tissues was moderate. In the present study, 35% of the samples had SP levels below the detection limit of ELISA. This may partly be due to having many sites in the present study slightly involved in periodontal inflammation. The SP level was also significantly correlated with indicators of host response. The results of Hanioka and colleagues showed that SP level in GCF may have a potential as an indicator of periodontal inflammation and the host response. Awawdeh and colleagues [21] examined a group consisting of 54 subjects, who had been diagnosed with irreversible pulpitis against one or more elements. This was the first study to quantify neuropeptides in GCF comparing painful teeth and the healthy contralateral. No teeth with pocket probing depths of more than 3 mm were included. Gingival crevicular fluid was collected from the mesial interproximal gingival crevice of each tooth diagnosed with irreversible pulpitis and scheduled to receive endodontic therapy. Significantly more of SP values were detected in GCF test element than the contralateral control element. After endodontic medication, the amount of SP decreased in 17 (81%) sites, it remained the same in a single site, and it was slightly increased in three (14%) sites. One week after pulp removal, there was no measurable SP in the GCF from seven (33%) initially painful teeth. The concentration of SP also decreased as a result of treatment. In contrast, the amount and concentration of SP in GCF from contralateral and adjacent teeth did not change significantly following pulp removal from the painful tooth. The presence of SP and NKA in GCF of painful and non-painful teeth raises the question of their origin. It is possible that the increased release of the tachykinins from peptidergic nerve endings in the inflamed dental pulp is mirrored by an increase in activity of similar fibres in the periodontium. This could result in higher concentrations of neuropeptides in the GCF not only from painful teeth but also from adjacent teeth. A significant decrease was found in the levels of SP in GCF after pulp removal, while no difference was evident in the contralateral elements. The authors explained the results saying that there are increases in neuropeptide levels, particularly of the tachykinins SP and NKA, in GCF associated with irreversible pulpitis in painful human teeth. Furthermore, there was a marked decrease in SP levels after pulp removal. At present, it is not possible to explain the exact mechanisms responsible for the high levels of neuropeptides in GCF in painful teeth.

## 5. Conclusions

During the literature analysis we have realized that several different basal levels of SP have been detected and this makes it difficult to compare the results obtained. However despite this limitation, it can be affirmed that in the crevicular fluid elements undergoing orthodontic force an appreciable amount of SP is present, while its level in control subjects cannot often be evaluated. Whereas the involvement of SP in periodontitis and inflammatory diseases is now well accepted, further studies are needed in order to demonstrate the role of this neuropeptide during teeth movement.

## Figures and Tables

**Figure 1:** Invisalign ClinCheck allows to predict dental movement with a very high precision, comparing every single element. This is an example of drowning: the first premolar coloured in blue is the control site and the second premolar is the test site. The blue color represents the position of the tooth before movement and the white one is the element subjected to dental flaring.

**Figure 2:** The picture shows the flaring movement in a lower incisor.

**Figure 3:** Example of drawings in the first upper premolar. The lips were moved with a cotton wool roll. Probing depth was collected with a paper cone from the mesial portion of the teeth.

**Table 1:** SP levels in crevicular gengival fluid of four patients. In the column on the left side, we had specified the number of patient and the dental element number using the FDI system of nomenclature, “T”: test tooth, “C”: control site. In the right column, there is the SP measurement expressed in pg.

Dental element	Measure (pg)
PZ.1 31 C	5.4
PZ.1 32 T	16.4
PZ.1 42 C	4.2
PZ.1 41 T	11.0
PZ.2 14 C	4.4
PZ.2 24 T	5.7
PZ.2 15 C	4.7
PZ.2 25 T	3.9
PZ.2 46 C	4.0
PZ.2 36 T	13.8
PZ.2 45 C	3.5
PZ.2 34 T	18.8
PZ.3 26 C	3.4
PZ.3 16 T	25.1
PZ.4 31 C	3.9
PZ.4 32 T	12.2
